# LncRNA AK045171 protects the heart from cardiac hypertrophy by regulating the SP1/MG53 signalling pathway

**DOI:** 10.18632/aging.102668

**Published:** 2020-02-21

**Authors:** Li Xu, Hongjiang Wang, Feng Jiang, Hao Sun, Dapeng Zhang

**Affiliations:** 1 Heart Center and Beijing Key Laboratory of Hypertension, Beijing Chaoyang Hospital, Capital Medical University, Beijing 100020, China

**Keywords:** LncRNA, cardiac hypertrophy, SP1/MG53

## Abstract

Hearts often undergo abnormal remodelling and hypertrophic growth in response to pathological stress. Long non-coding RNAs (LncRNAs) can change cardiac function and participate in regulation of cardiac hypertrophy. The present study aims to identify the role of AK045171 in cardiac hypertrophy and the underlying mechanism in hypertrophic cascades. Mice with cardiac hypertrophy were established through transverse aortic constriction (TAC). Cardiac hypertrophy in cardiomyocytes was induced by angiotensin II (angII). The expression of AK045171 and its target gene SP1 was examined in cardiomyocytes transfected with miRNA. The AK045171 expression level was downregulated in mice after TAC surgery. Overexpression of AK045171 attenuated cardiac hypertrophy both in vitro and in vivo. The mechanism study indicated that AK045171 binds with SP1, which promotes transcription activation of MEG3. It is suggested that overexpression of AK045171 might have clinical potential to suppress cardiac hypertrophy and heart failure.

## INTRODUCTION

Mechanical stress or neurohormonal stimulation, including hypertension, ischaemia and myocarditis, induce cardiac hypertrophy, which is characterized by an increase in cardiomyocyte size without a change in cell number [1]. Sustained hypertrophy can change the deposition of extracellular collagen, induce a loss of adrenergic responsivity and alter cell metabolism, making it one of the most important risk factors for heart failure and sudden death [2, 3]. Understanding the molecular mechanisms underlying hypertrophy initiation and progression will aid in developing novel and effective therapeutics for hypertrophy.

Recently, despite the numerous genes and proteins that have been demonstrated to participate in the modulation associated with cardiac hypertrophy, the mechanisms remain incompletely understood.

Non-coding RNAs (ncRNAs) account for approximately 98% of the entire human genome. Long non-coding RNAs (LncRNAs) are a novel group of ncRNAs with a length of more than 200 nucleotides [4]. LncRNAs are capable of regulating gene expression at epigenetic, transcriptional and post-transcriptional levels and thus participate in various of pathological processes, such as autophagy, necrosis, and apoptosis, which can lead to myocardial hypertrophy or cardiac remodelling [5–7].

Increasing evidence has demonstrated the crucial role of lncRNAs in both the development and pathology of the cardiovascular system, including cardiac hypertrophy. For instance, Chaer (Cardiac Hypertrophy-Associated Epigenetic Regulator) contributes to progression of cardiac hypertrophy by directly interacting with the catalytic subunit of polysome repressor complex 2 (PRC2), thereby inhibiting histone H3 lysine 27 methylation at the promoter region of genes involved in cardiac hypertrophy [8]. Mhrt binds with the histone acetylation factor Brg1 and further antagonizes the function of Brg1, which is activated by stress as a chromatin-remodelling factor to trigger aberrant gene expression and cardiomyopathies [9, 10]. Chast induces cardiomyocyte autophagy and drives hypertrophy by inhibiting Plekhm1 expression [11]. In addition to their gene- or chromatin- regulation effect, lncRNAs also function as sponges of miRNAs. For instance, CHRF, ROR, H19, and MIAT are involved in hypertrophy progression through sponging of miR-489 [12], miR-133 [13], miR-675 [14] and miR-150 [15], respectively. Although many studies on the role of lncRNAs in cardiac hypertrophy have been conducted and the mechanism has been partially identified, further research should be conducted.

In this study, we aimed to determine the function of the novel lncRNA AK045171 in hypertrophy, which has not been previously elucidated. Down-regulation of AK045171 expression in hypertrophic cardiomyocytes was confirmed. Function studies revealed that AK045171 was capable of inhibiting hypertrophy progression and cardiac fibroblast activation. In addition, we found that AK045171 binds to SP1, which is a critical transcription factor that regulates the transcription of MG53 and its downstream signalling pathways, such as GSK-3β/β-catenin and NF-ΚB. These findings offer important insights into fundamental mechanisms underlying lncRNA function as well as a novel therapy venue for cardiac hypertrophy and its underlying pathology.

## RESULTS

### AK045171 was down-regulated in myocardium from mice that underwent TAC and in cardiomyocytes treated with angiotensin II

We first established an in vivo hypertrophy model via a TAC operation and an in vitro model via treatment of cardiomyocytes with angiotensin II for further research. The results showed that hearts from TAC-treated mice were larger than those from normal mice; in addition, individual cardiomyocytes in the TAC group were accordingly larger (Figure 1A). Echocardiographic parameters of the mice, including LVEDP, LVFS, LVEF, and LVESD, were evaluated with an ultrasound system and further indicated that cardiac function in the mice subjected to TAC was impaired (Figure 1B, 1C). Masson staining revealed that the TAC surgery induced significant myocardial fibrosis (Figure 1E). α-SMA staining of cardiomyocytes was carried out to detect their size after ang II treatment. Obviously, ang II increased cardiomyocyte size compared with normal cells (Figure 1F). The levels of ANP, BNP and β-MHC are typically used to evaluate the extent of myocardial hypertrophy, and their levels in the Ang II treatment group were found to be elevated (Figure 1G). To detect the expression level ofAK045171 in cardiac tissues from mice with cardiac hypertrophy, we measured the expression level via quantitative real-time PCR in tissues from the left ventricle of mice in the cardiac hypertrophy and sham groups. AK045171 expression was downregulated in the myocardium with cardiac hypertrophy compared with that in sham group mice, which is consistent with the heart weight to tibial length ratio (HW/TL) (Figure 1H). Similarly, AK045171 expression was decreased in cardiomyocytes after ang II treatment compared with that in normal cells (Figure 1I).

**Figure 1:** **AK045171 was downregulated in cardiomyocytes and myocardium subjected to AngII and TAC treatment.** (**A**) Haematoxylin and eosin staining of the heart under sham and TAC treatment to investigate the size of the heart and cardiomyocytes. (**B**, **C**) Echocardiographic parameters of the mice, including LVEDP, LVFS, LVEF, LVESD, were evaluated with an ultrasound system. (**D**) Quantification of the heart weight-to-tibial length ratio. (**E**) Masson staining was used to detect myocardial fibrosis. (**F**) Immunostaining for α-SMA was used to evaluate the size of cardiomyocytes subjected to AngII treatment or not. (**G**) The level of the myocardial hypertrophy biomarkers ANP, BNP and β-MHC were detected using qPCR. (**H**, **I**) The expression of AK045171 was detected with qPCR. *p<0.05 vs control or sham group.

### Overexpression of AK045171 suppressed cardiac hypertrophy both in vitro and in vivo

To identify whether AK045171 protects cardiomyocytes from stimulus-induced hypertrophy, cardiomyocytes were transduced with adenovirus vector containing an AK045171 overexpression vector. To detect the efficiency of the adenovirus, we evaluated the expression of AK045171 in each group, and the results indicated that the AK045171 adenovirus significantly elevated the expression level of AK045171 both in vivo and in vitro compared with that in the anti-NC group (Figure 2A, 2B).

**Figure 2:** **AK045171 ameliorated the hypertrophy in vitro and in vivo induced by AngII and TAC treatment.** (**A**, **B**) qPCR was used to evaluate the efficiency of AK045171overexpression adenovirus, which significantly elevated the level of AK045171 in cardiomyocytes and myocardium. (**C**) Echocardiographic parameters of the mice, including LVEDP, LVFS, LVEF, and LVESD, were evaluated with an ultrasound system. (**C**) Haematoxylin and eosin staining of the heart under TAC, TAC+Ad-AK045171 or TAC+ Ad-vector treatment. (**D**) Quantification of heart weight-to-tibial length ratio. (**E**) Immunostaining of α-SMA was used to evaluate the size of cardiomyocytes subjected to AngII, AngII+ Ad-AK045171 or AngII+Ad-vector treatment. (**F**) The level of the myocardial hypertrophy biomarkers ANP, BNP and β-MHC were detected using qPCR. * p<0.05 vs the Ang II+Ad-vector or TAC+Ad-vector group.

To elucidate whether AK045171 was capable of decreasing cardiac hypertrophy in vivo, mice were injected with Ad-AK045171 in the heart 1 week after TAC surgery. TAC-induced cardiac hypertrophy in mice was expected to be reflected by increased heart weight, and Ad-AK045171 overexpression in mice reversed the TAC-induced changes. Cardiomyocyte size was determined in histological sections of hearts and was found to be significantly decreased in the Ad-AK045171 group compared with the Ad-vector group (Figure 2B). To assess cardiac function, the parameters LVEDP, LVFS, LVEF, and LVESD were detected. LVEDP and LVESD were significantly reduced in the Ad-AK045171 group compared with the Ad-vector group. LVFS and LVEF were significantly improved in the Ad-AK045171 group at 4 weeks (Figure 2C).

In response to Ang II treatment, the average cardiomyocyte size was decreased in the Ad-AK045171 group compared with the Ad-vector control group, suggesting that excessive AK045171 expression restored the cardiomyocyte phenotype under stimulation with Ang II (Figure 2E). Moreover, AK045171 overexpression significantly reduced the expression levels of ANP, BNP and β-MHC compared with those in the anti-NC group (Figure 2F), consistent with the heart weight to tibial length ratio (HW/TL) (Figure 2D).

Taken together, these results demonstrate that overexpression of AK045171 can protect the heart from cardiac hypertrophy both in vitro and in vivo.

### AK045171binds to SP1 and promotes the expression of MG53

It is well known that lncRNA is capable of binding to DNA or mRNA and regulating gene transcription or translation. To explore the mechanism underlying the effect of AK045171in cardiac hypertrophy, we carried out RNA pull-down and silver staining assays. We found a specific band at 72 kDa, and the results of further mass spectrometry analysis suggested that AK045171may interact with SP1, which is a critical transcription factor (Figure 3A). To validate this prediction, we conducted RNA pull-down and RIP assays. As expected, the results indicated that AK045171 specifically binds to SP1 (Figure 3B, 3C). As we know, SP1 is a transcription factor that is primarily localized in the nucleus and plays various roles by modifying the transcription of target genes. We wondered whether AK045171 is also localized in the cell nucleus. qPCR and FISH experiments confirmed our speculation. AK045171 primarily exists in the nucleus, similar to SP1 (Figure 3D, 3F). AK045171 has a length of more than 2000 nucleotides. We divided the entire sequence into four parts to further discover which portion of the sequence interacts with SP1. The results revealed that the 1-500-bp region of AK045171 is the region that binds to SP1 (Figure 3G).

**Figure 3:** **AK045171 binds to SP1 and regulates the expression of MG53.** (**A**) RNA pull-down and silver staining assays were performed to investigate the potential proteins that combined with AK045171. (**B**) RNA pull-down and (**C**) RIP assays were used to confirm the interaction between AK045171 and SP1. (**D**) We next evaluated the location of AK045171 in cardiomyocytes and found that AK045171 primarily exists in the cell nucleus. (**E**, **F**). Immunofluorescence was used to further detect the expression and location of AK045171. (**G**) The entire sequence of AK045171 was divided into 4 sections to determine which region binds with SP1 using an RNA pull-down assay. (**H**, **I**) Luciferase activity assays were performed to detect whether knockdown or overexpression of AK045171 influences SP1 transcription. (**J**) ChIP assay was used to determine the binding of SP1 and the promoter of MG53 after AK045171 knock down. (**K**) Western blot was used to detect the expression of MG53 under AK045171 overexpression or knock down. (**L**) Evaluation of the MG53 protein level after SP1 deletion with a Crispr/cas9 system. *p<0.05 vs the IgG, si-control, Ad-vector or wt group; ^#^ p<0.05 vs Ad-vector group.

SP1 is well known to be a critical transcription factor that participates in regulation of various important genes involved in biological processes. We were curious about the target genes of SP1 through which it may target and change the phenotype of cardiomyocytes. Bioinformatic analysis software was used to predict the potential target genes of SP1. Among the genes identified, MG53 attracted our attention because of the crucial role it plays in the development of cardiovascular disease, such as ischaemia-reperfusion injury and hypertrophy. To confirm our speculation, we performed a luciferase activity assay. As shown in Figure 3H and 3I, deletion of AK045171 using three siRNA inhibited the luciferase activity of MG53. In contrast, overexpression of AK045171 through Ad-AK045171 promoted the luciferase activity of the MG53 gene. ChIP assay revealed that AK045171 knock down inhibited the binding of SP1 to the promoter of MG53 (Figure 3J). Detection of the MG53 protein level further revealed that deletion of AK045171 inhibited while overexpression of AK045171 promoted MG53 protein expression (Figure 3K). Moreover, we deleted the SP1 using CRISPR/Cas9 system. The results indicated that SP1 was effectively knock out. And SP1 knock out significantly inhibited the expression of MG53 (Figure 3L).

### AK045171 regulates the MG53/GSK3/β-catenin and MG53/NFκB pathways

MG53 is an extremely important cardiac-specific transcription factor that has been reported to be involved in regulation of the GSK3/β-catenin and NFκB signalling pathways. We sought to determine whether AK04517 is involved in regulation of the GSK3/β-catenin and NFκB signalling pathways through MG53. Western blotting was conducted to evaluate the protein expression level of relevant genes. The results showed that AK045171 promoted the expression of MG53 and the phosphorylation of β-catenin, which decreased translocation of β-catenin into the nucleus. The expression of the hypertrophy biomarkers ANP, BNP and β-MHC may be altered by the level of the transcription factors β-catenin or NFκB (Figure 4A, 4B). Moreover, we found that AK045171 was capable of inhibiting IKKβ and IκBα phosphorylation, which further inhibited translocation of p65 into the nucleus (Figure 4C–4E).

**Figure 4:** **AK045171 is involved in the regulation of MG53/GSK3/β-catenin and MG53/NFκB pathways.** Western blotting was used to evaluate the expression levels of proteins in the MG53/GSK3/β-catenin (**A**, **B**) and MG53/NFκB (**C**, **D**) pathways. (**E**) Immunofluorescence staining of p65 was performed to observe nuclear transfer of p65. * p<0.05 vs Ad-vector group; # p<0.05 vs Ad-AK054171+si-nc group.

### Knockdown of MG53 reversed the effect of AK045171 on cardiac hypertrophy

We further evaluated the role of MG53 in cardiac hypertrophy and its interaction with AK045171 using rescue experiments. A qPCR assay was used to evaluate MG53 and AK045171 expression. The results revealed a significantly elevated level of AK045171 in cardiomyocytes after infection with Ad-AK045171, but knockdown of MG53 did not influence the expression of AK045171. Moreover, Ad-AK045171 notably promoted the level of MG53, while MG53 deletion significantly inhibited the level of MG53 compared with that in the AK045171 overexpression group (Figure 5A, 5B). Knockdown of MG53 partially increased cardiac hypertrophic growth, which was inhibited by AK045171 overexpression (Figure 5C–5F). Like in the in vivo experiments, qPCR results revealed a significantly elevated level of AK045171 in cardiomyocytes after infection with Ad-AK045171, but knockdown of MG53 did not influence the expression of AK045171. (Figure 5G, 5H). Assessment of cardiomyocyte size and the expression of hypertrophic genes, including ANP, BNP and β-MHC, demonstrated that MG53 knockdown reversed the protective effect of AK045171 on cardiac hypertrophy induced by Ang II treatment (Figure 5I, 5J).

**Figure 5:** **MG53 knockdown reversed the effect of AK045171 on cardiac hypertrophy.** (**A**, **B**) qPCR was used to evaluate the efficiency of adenoviruses used to induce AK045171 overexpression or knockdown in myocardium and the expression of MG53. (**C**, **D**) HE staining of the heart under TAC, TAC+Ad-AK045171, TAC+ shRNA and TAC+sh-MG53 treatment. TAC significantly elevated the level of AK045171 in cardiomyocytes and myocardium. (**E**) The echoradiographic parameters LVEDP, LVFS, LVEF, and LVESD in mice were evaluated with an ultrasound system. (**F**) Quantification of heart weight-to-tibial length ratio. (**G**, **H**) qPCR was used to evaluate the efficiency of adenoviruses used for AK045171 overexpression and knockdown in cultured cardiomyocytes and the expression of MG53 (**I**) The level of the myocardial hypertrophy biomarkers ANP, BNP and β-MHC were detected using qPCR. (**J**) Immunostaining of α-SMA was used to evaluate the size of cardiomyocytes subjected to AngII, AngII+Ad-AK045171, AngII+Ad-AK045171+shRNA or AngII+Ad-AK045171+sh-MG53 treatment.*p<0.05 vs TAC or Ang II group; ^#^ p<0.05 vs TAC+Ad-AK054171+si-nc or Ang II+Ad-AK054171+si-nc group.

### AK045171 inhibited cardiac fibroblast proliferation

Cardiac fibroblasts play critical roles in myocardial hypertrophy. Thus, we next explored whether AK045171 is involved in alteration of cardiac fibroblasts. Cell proliferation and the expression of activation biomarkers, including collagen I, collagen III and MMP9, were evaluated. The MTT (Figure 6A) and EDU (Figure 6B) staining results suggested that AK045171 notably inhibited the cell proliferation that was promoted by MS treatment. Moreover, qPCR (Figure 6C–6E) and Western blotting (Figure 6F) was used to detect the level of collagen I, collagen III and MMP9 and demonstrated that AK045171 significantly decreased the collagen I, collagen III and MMP9 expression levels, which indicated that AK045171 is capable of inhibiting the activation of cardiac fibroblasts. Figure 7 showed the molecular mechanism underlying the effect of AK045171 in TAC- and Ang II-induced cardiac hypertrophy.

**Figure 6:** **AK045171 inhibited the proliferation of cardiac fibroblasts.** (**A**) MTT assays were used to evaluate cardiac fibroblast proliferation. (**B**) EDU staining was performed to detect the proliferation of cardiac fibroblasts. qPCR was used to detect the expression of fibrosis biomarkers, including (**C**) collagen I (**D**) collagen III and (**E**) MMP-9. (**F**) Western blotting was carried out to investigate collagen I, collagen III and MMP-9 protein expression. *p<0.05 vs control group; ^#^p<0.05 vs MS+vector group.

**Figure 7:** **Schematic showing the possible molecular mechanism underlying the effect of AK045171 in TAC- and Ang II-induced cardiac hypertrophy.** AK045171 binds with SP1 and activates MG53 transcription. MG53 inhibits nuclear transfer of p65 and β-catenin, thereby decreasing expression of their downstream target genes, such as ANP, BNP and β-MHC.

## DISCUSSION

Previous studies have demonstrated that lncRNAs are correlated with cardiac diseases; however, research focused on the effect of lncRNAs in cardiac hypertrophy is still relatively rare. In the present study, we identified and confirmed that AK045171expression is downregulated. Further in vivo and in vitro function studies demonstrated that AK045171 overexpression significantly suppressed cardiac hypertrophy and activation of cardiac fibrosis. Moreover, AK045171 binds SP1 and participates in transcriptional regulation of MG53, thereby changing the expression of factors in downstream signalling pathways involved in hypertrophy progression.

Sp1 is a ubiquitously expressed, prototypic C2H2-type, zinc finger-containing DNA binding protein that can activate or repress transcription in response to physiologic and pathological stimuli [16–18]. It binds GC-rich motifs with high affinity and can regulate the expression of TATA-containing and TATA-less genes via protein-protein interactions or interplay with other transcription factors [19, 20], such as Ets-19582348 [21], c-myc [22], c-Jun(1972), Stat1 [23] and Egr-1 [24]. Recent studies have also consistently demonstrated elevations in SP1 levels in cardiac hypertrophy result from increased left-rights hunting, volume loading of the left ventricle, pressure loading of the right ventricle, or angiotensin II stimulation [25, 26]. Moreover, gentisic acid has been reported to attenuate cardiac hypertrophy and fibrosis through downregulation of Sp1/GATA4 signalling [27]. Another report showed that Sp1 could be recruited to the ANF promoter, which is a cardiac gene, and that GATA4 could cooperate with Sp1 to activate ANF transcription; moreover, a direct interaction between GATA4 and Sp1 was observed [28]. We performed a bioinformatic analysis using AnimalTFDB3.0 to predict the target genes of SP1 and interestingly found that MG53 was a predicted target gene; MG53 has recently attracted the attention of scientists due to its crucial role in cardiovascular disease. MG53 is an essential component of the membrane repair machinery in striated muscles [29, 30]. In a recent study, MG53 mRNA levels were demonstrated to be decreased in PE-stimulated cardiomyocyte hypertrophy and TAC-induced cardiac hypertrophy, which is consistent with our findings [31].

Herein, we first confirmed that AK045171lncRNA directly interacts with SP1 and that SP1 is capable of activating MG53transcription. Interestingly, AK045171lncRNA promoted the expression of MG53.

Furthermore, we aimed to explore the downstream genes of SP1/MG53 signaling. MG53 contributes to cardiac fibrosis by regulating STAT3/Notch-1 signalling [32]. It can also negatively regulate myogenesis by targeting insulin receptor substrate 1 and PPAR-α expression at the transcriptional level to induce diabetic cardiomyopathy [33]. MG53 exerts a cardioprotective effect during ischaemia-reperfusion injury through phosphorylation of GSK-3 [14, 34], and because ischaemia-reperfusion injury is also a risk factor for sudden cardiac death and heart failure and post-MI cardiac hypertrophy, MG53 has emerged as a promising target in the treatment of MI patients. In addition, heterozygous deletion of β-catenin in a pressure overload mouse model induced significant upregulation of the foetal gene programme—β-myosin heavy chain and atrial and brain natriuretic peptides (ANP and BNP). We speculated that an interaction between MG53 and GSK-3 is possible. Therefore, MG53 might promote the expression of GSK-3 and phosphorylation of β-catenin [35].

Next, because MG53 has been demonstrated to regulate KChIP2 and Ito,f by modulating NF-κB activity, we further evaluated whether there were any alterations in the NF-κB pathway. Interestingly, MG53 inhibited the phosphorylation of IKKβ and IκB-α, thereby attenuating transportation of p65 into the nucleus. It is well known that NF-κB (p65) can inhibit myocardin- induced cardiomyocyte hypertrophy through multiple mechanisms. Thus, p65 may be another downstream gene under control of MG53 in cardiac hypertrophy. Both the GSK-3β/β-catenin and NF-ΚB pathway are involved in regulation of cardiac genes, such as ANP, BNP and β-MHC. However, we did not confirm whether SP1/MG53 directly modifies the expression of ANP, BNP and β-MHC through the GSK-3β/β-catenin and NF-ΚB pathways or indirectly through other signalling pathways. In addition, MG53 has been reported to be an endogenous regulator of cardiac KChIP2 expression and Ito,f by regulating the NF-κB signalling pathway, thus playing an important role in maintaining cardiac electrical stability in hypertrophy. However, it was reported by Caimei Zhang et al. that MG53 is upregulated upon chronic pathological cardiac stress, such as in pressure overload-induced hypertrophy and heart failure [36]. We tried to find an explanation for these results and found another study indicating that when TRIM72 is highly and continuously expressed, IRS-1 level is decreased and AKT signalling is down-regulated. These activities lead to a decrease in heart size. However, a compensatory mechanism must exist to block this reduction in heart size [37]). MG53 transcriptionally upregulates peroxisome proliferation-activated receptor alpha and its target genes, resulting in diabetic cardiomyopathy, indicating complicated mechanisms underlying its biological effects [38]. Clarifying the complicated mechanism underlying the effect of MG53 in initiation or progression of cardiac hypertrophy still needs much work. This work will be performed in our future studies.

In conclusion, we revealed that lncRNA plays a critical role in the development of cardiac hypertrophy. It was first demonstrated that lncRNA interacts with SP1, primarily in the nucleus, and promotes transcription of the MG53 gene. Further molecular mechanistic study indicated that MG53 participates in regulation of the GSK-3β/β-catenin and NF-ΚB signalling pathways.

In this study, we extended the understanding of the role of lncRNA in cardiac hypertrophy and provided a novel regulatory mechanism underlying the effect of lncRNA and transcription factors, such as SP1 and MG53. Our findings suggest novel biomarkers or potential therapeutic targets to treat hypertrophy. The side effect of adenovirus on other organs remain unclear which will be evaluated in our future work. Moreover, elucidation of the deep regulatory relationship between these molecules also requires further studies.

## MATERIALS AND METHODS

### Transverse aortic constriction (TAC)

90 C57BL/6 mice obtained from Beijing Vital River laboratory animal center were transduced with different kinds of genes and subjected to transverse aortic constriction procedure Briefly, mice weighing 25-30 g (8 weeks) were anaesthetized with isoflurane and subjected to thoracotomy. The aorta was dissected and tied with a 7-0 silk thread around the vessel using a 26-gauge needle to ensure consistent occlusion. Mice in the sham group underwent thoracotomy and aortic dissection without constriction of the aorta. All the animal procedures were performed in accordance with the guidelines of Capital Medical University Animal Care and Use Committee.

### Adenovirus application in TAC models

Adenoviruses to induce AK045171 overexpression or MG53 knockdown and their negative controls were designed and synthesized by Hanbio (Tianjin, China). These adenoviruses alone or together were injected into mice in the heart 1 week before the TAC operation (3.5×10^7^ viral particles). Four weeks after the TAC operation, the hearts were collected, and the left ventricle was rapidly frozen in liquid nitrogen and stored at −80°C for subsequent experiments.

### Crispr/cas9 vector establishment

This plasmid contains two expression cassettes, hSpCas9 and the chimeric guide RNA. The vector was designed (sgSP1 forward: CACCGTCATTCGGACA CCAACCGTG; sgSP1 reverse: AAACCACGGTTGG TGTCCGAATGAC) which was annealed and digested using BsmBI. The oligos were cloned into the single guide RNA scaffold lentiCRISPRv2 vector.

### Echocardiography in mice

Echocardiography was performed using a Visualsonics Vevo 2100 ultrasound system Toronto, Canada) with a 40-MHz transducer. Left ventricular end-systolic diameter (LVESD) and left ventricular end-diastolic pressure (LVEDP) were measured. Percent left ventricular fractional shortening (LVFS) and left ventricular ejection fraction (LVEF) were calculated according to the system.

### Cardiomyocyte and cardiac fibroblast culture and transduction

Neonatal mouse cardiomyocytes and cardiac fibroblasts were isolated from the heart of newborn C57BL6 mice (1day old). Briefly, the mice were anaesthetized and sacrificed by immersion into 75% (v/v) alcohol. After thoracotomy, the hearts were exposed and quickly excised. The ventricles were isolated and transferred into cold Hank’s balanced salt solution (HBSS; Invitrogen, CA, USA) without Ca^2+^ or Mg^2+^. The tissue was dispersed through a series of incubations at 37°C in HBSS containing 1.2 mg/ml pancreatin and 0.14 mg/ml collagenase. After centrifugation, cells were resuspended in Dulbecco’s modified Eagle’s medium (DMEM; Invitrogen, CA, USA) containing 20% foetal bovine serum (FBS; Invitrogen, CA, USA) and supplemented with antibiotics (penicillin, streptomycin; Invitrogen, CA, USA). Thereafter, cells were seeded and cultured at 37 °C in a humidified atmosphere of 95% air and 5% CO_2_. After 2 h, the supernatant was transferred into a new culture flask together with cells that were not attached, indicating that they were cardiomyocytes. The attached cells were maintained as cardiac fibroblast cells. For transduction, the cells were plated in a 6-well plate at a density of 2×10^5^ cells per well. After 24 h of culture, the cells were transduced with adenovirus to induce AK045171 overexpression or MG53 knockdown as well as with their negative controls at 2×10^5^ viral particles/ml. Twelve hours after transduction, the medium was replaced with serum-free medium. and the cells were incubated for an additional 48 hours in 1 μM Angiotensin II (angII;Sigma, CA, USA) for further study.

### Mechanical stretching (MS)

Mechanical stretching was performed on flexible silicon membranes. In brief, cardiac fibroblasts were plated at a density of 4×105 cells/ml on BioFlex culture plates coated with Collagen I. When the cell confluent reach to 70%, the culture medium was replaced by serum free medium before stretching. Culture plates were mounted on the Baseplate™ and cyclic stretch was applied in the FX-4000T™ Tension Plus™ System (Hillsborough, USA) with 20% elongation, 0.5 Hz in a half sinus regimen [39].

### Quantitative real-time PCR (qRT-PCR)

Total RNA from heart tissue or cardiomyocyte cultures was extracted according to the TRIzol (Invitrogen, CA, USA) instructions, and the concentration and purity of RNA were detected using an ultramicro spectrophotometer (NanoDrop, Thermo, USA). For reverse transcription, the RNA was reversely transcribed to cDNA in a total system of 20 μl. Reverse transcription was performed at 25°C for 5 min followed by 50°C for 45 min and inactivation of the reverse transcriptase at 85°C for 5 min. The cDNA was synthesized and analysed via qRT-PCR, and qRT-PCR was conducted in accordance with the instructions of a SYBR Premix Ex Taq™ II reagent kit (Takara, Dalian, China). The mRNA level of target genes was normalized to GAPDH gene expression. The gene expression levels of ANP, BNP and β-MHC in cardiomyocytes treated with ang II were determined via real-time quantitative RT-PCR using the 2^−ΔΔCt^ method.

### MTT

After transfection, 6×10^3^ cardiac fibroblasts/well were seeded into 96-well plates. Following culture for 24 h, 0.5% MTT (Beyotime, Shanghai, China) was added to the culture medium and incubated with the cells for 4 h. Subsequently, the culture medium was removed, and DMSO was added into each well. After that, the absorption at 490 nm was evaluated using a microplate reader (Bio-Rad, USA).

### EDU staining

Cardiac fibroblasts were fixed in 4% paraformaldehyde for 30 min at room temperature. Next, 1%TritonX-100A was added for permeabilization, and the cells were incubated with an EdU reaction cocktail (Click-iT EdU Microplate Assay Kit, USA) for 30 min following the instructions. Finally, cellnuclei were stained with 1 mg/ml DAPI (Beyotime, Shanghai, China) for 15 min, and the cells were observed under a fluorescence microscope (Leica, Wetzlar, Germany).

### Immunostaining

For immunostaining, cells were fixed with 4% paraformaldehyde for 20 min, permeabilized with 0.5% Triton X-100 for 15 min, and then blocked with 3% BSA for 30 min. The cells were incubated with the indicated primary antibody (α-SMA; Abcam, Cambridge, England) at 4 °C overnight. After 3 washes, the cells were incubated with Alexa Fluor-labelled secondary antibody (Invitrogen, CA, USA) for 2 h followed by DAPI (Beyotime, Shanghai, China) staining for another 10 min (Olympus, Japan).

### Histology assay

Heart tissue samples from mice were collected at 4 weeks after TAC. The specimens were fixed with 4% paraformaldehyde, embedded in paraffin, cut into 5-μm-thick sections and stained with haematoxylin and eosin (HE) according to the manufacturer’s instructions.

### Western blot analysis

Samples were lysed in RIPA lysis buffer containing protease inhibitor cocktail (Beyotime, Shanghai, China) on ice for 30 min and centrifuged at 12,000×g for 15 min at 4°C. The nuclear protein was extracted using a nuclear and cytoplasmic protein extraction kit (Beyotime, Shanghai, China). The supernatants were collected and stored at -80°C. The protein concentrations were measured using a BCA Protein Assay Kit (Beyotime, Shanghai, China) according to the manufacturer’s protocol. The tissue or cell extracts were subjected to SDS-PAGE and Western blot analysis. Proteins blotted on PVDF membranes were incubated with primary antibodies overnight at 4°C. Goat anti-mouse (1:2,000) or anti-rabbit (1:2,000) secondary antibodies (Abcam, DC, USA life) were then utilized. The protein bands were visualized using a chemiluminescence imaging system (Tannon, Shanghai, China).

### Fluorescence in situ hybridization (FISH)

Alexa Fluor 555-labelled AK045171 probeswas designed and synthesized by RiboBio (Guangzhou, China). FISH experiments were carried out with a Fluorescence In Situ Hybridization Kit (RiboBio, Guangzhou, China). Cells (1×10^5^) were seeded onto autoclaved glass slides and cultured for 24 h. After fixation with 4% paraformaldehyde for 20 min followed by permeabilization with 0.5% Triton X-100 for 10 min, the cells were cultured at 37°C overnight. Finally, the slides were incubated with DAPI to stain cell nuclei and observed under a fluorescence microscope (Leica, Wetzlar, Germany).

### RNA pull-down assay

A biotin-labelled AK045171 probe and control probe were synthesized by Sangon Biotech (Shanghai, China). Probe-coated beads were generated by co-incubation of the probe with streptavidin-coated beads (Invitrogen, CA, USA) at 25°C for 2 h. Cardiomyocytes were collected, lysed and incubated with the AK045171 probes overnight at 4°C. Thereafter, the beads were eluted, and the complex was purified with TRIzol (Takara, Dalian, China). Then, the abundance of SP1 was analysed via western blot.

### Luciferase reporter assay

The promoter sequence of MG53 was inserted into the pGL3 vector and generate recombinant plasmids. Subsequently, the plasmids were transformed into cardiomyocytes along with siRNA or overexpressing plasmids of AK045171. A luciferase assay was performed using the Dual-Luciferase Reporter Assay System (Promega, USA) on a GloMax 20/20 Luminometer (Promega, USA) according to the manufacturer’s instructions.

### Chromatin immunoprecipitation (ChIP) assay

Cells were fixed using formaldehyde solution for the preparation DNA-protein cross-link. Chromatin fragments were obtained by application of ultrasonic sound (10 seconds each time at an interval of 10 seconds, 12 times). The supernatant was collected through centrifugation at 12000g and 4°C for 10 minutes. Thereafter, the supernatant was incubated with antibody to IgG or antibody to SP1 at 4°C overnight. The DNA-protein complex was precipitated using protein agarose/sepharose, followed by centrifugation at 16099g for 5 minutes. The supernatant was discarded, and the non-specific complex was washed. De-cross-linking was conducted at 65°C overnight. DNA fragment was purified and extracted using phenol/chloroform. The binding of SP1 to the MG53 promoter was determined by RT-qPCR.

### Statistical analysis

All data are presented as the mean ± standard deviation (SD) of at least three repeated individual experiments and were analysed using GraphPad Prism version 5.00 software (GraphPad, CA, USA). Statistical significance was determined with an unpaired two-tailed Student t test (for two groups). A value of p<0.05 was considered statistically significant.
